# Efficacy of Whole-Body Vibration Training on Brain-Derived Neurotrophic Factor, Clinical and Functional Outcomes, and Quality of Life in Women with Fibromyalgia Syndrome: A Randomized Controlled Trial

**DOI:** 10.1155/2021/7593802

**Published:** 2021-11-30

**Authors:** Vanessa G. C. Ribeiro, Ana C. R. Lacerda, Jousielle M. Santos, Ana C. Coelho-Oliveira, Sueli F. Fonseca, Ana C. N. Prates, Jurandir Flor, Bruna C. C. Garcia, Rosalina Tossige-Gomes, Hércules R. Leite, José S. C. Fernandes, Arthur N. Arrieiro, Alessandro Sartorio, Borja Sañudo, Danubia C. Sá-Caputo, Mário Bernardo-Filho, Pedro H. S. Figueiredo, Henrique S. Costa, Vanessa P. Lima, Renato F. Cardoso, Alessandra C. Bastone, Luana A. Soares, Vanessa A. Mendonça, Redha Taiar

**Affiliations:** ^1^Integrated Center for Research and Post-Graduate Studies in Health (CIPq), Federal University of the Jequitinhonha and Mucuri Valleys (UFVJM), Diamantina, Minas Gerais, Brazil; ^2^Multicentric Postgraduate Program in Physiological Sciences (PPGMCF), Brazilian Society of Physiology, Diamantina, MG, Brazil; ^3^Physiotherapy Department, Faculty of Biological Sciences and Health, Federal University of the Jequitinhonha and Mucuri Valleys, Diamantina, MG, Brazil; ^4^Postgraduate Program in Functional Performance and Rehabilitation (PPGReab), Federal University of the Jequitinhonha and Mucuri Valleys, Diamantina, MG, Brazil; ^5^Postgraduate Program in Health Sciences (PPGCS), Federal University of the Jequitinhonha and Mucuri Valleys, Diamantina, MG, Brazil; ^6^Mechanical Vibration Laboratory and Integrative Practices (LAVIMPI), Biophysics and Biometrics Department, Institute of Biology Roberto Alcântara Gomes and Piquet Carneiro Polyclinic, Rio de Janeiro State University, Rio de Janeiro, Brazil; ^7^Postgraduate Program in Rehabilitation Sciences (PPGCR), School of Physical Education Physiotherapy and Occupational Therapy, Federal University of Minas Gerais, Belo Horizonte, MG, Brazil; ^8^Faculty of Agrarian Sciences, Federal University of the Jequitinhonha and Mucuri Valleys, Diamantina, MG, Brazil; ^9^Istituto Auxologico Italiano, Division of Metabolic Diseases and Auxology & Experimental Laboratory for Auxo-endocrinological Research, Verbania, Italy; ^10^Department of Physical Education and Sport, University of Seville, Seville 41013, Spain; ^11^MATériaux et Ingénierie Mécanique (MATIM), Université de Reims Champagne-Ardenne, Reims, France

## Abstract

This study aimed to investigate the efficacy of whole-body vibration training (WBVT) on blood brain-derived neurotrophic factor (BDNF) levels and determine the clinical and functional outcomes in patients with fibromyalgia syndrome (FMS). Thirty-two women with FMS were randomized into an intervention group (IG), receiving 6 weeks of WBVT, or a control group (CG) with no intervention. The outcomes at the baseline and follow-up in both groups included blood BDNF levels, sit-to-stand test (STS), 6-minute walk test (6MWT), Fibromyalgia Impact Questionnaire (FIQ), Pittsburgh Sleep Quality Index (PSQI), Beck Depression Inventory (BDI), and visual analogue scale (VAS). WBVT resulted in a group-by-time interaction effect. Thus, after the intervention time, the IG had increased blood BDNF levels (*p*=0.045), a higher number of repetitions on the STS test (*p*=0.011), and increased walking distance on the 6MWT (*p*=0.010), compared to CG. Moreover, there was a reduction in the scores of the FIQ (*p*=0.001), the PSQI (*p*=0.001), the BDI (*p*=0.017), and pain assessed using VAS (*p*=0.008) in IG. The results demonstrate that WBVT promotes an increase in blood BDNF levels, with concomitant improvement in lower limb muscle strength, aerobic capacity, clinical symptoms, and quality of life in women with FMS. This trial is registered with Brazilian Clinical Trials Registry (REBEC; RBR-38nbbx) (https://ensaiosclinicos.gov.br/rg/RBR-38nbbx).

## 1. Introduction

Fibromyalgia syndrome (FMS) is characterized by chronic widespread pain, neuroinflammation [1], nociception-driven amplification of neural signalling (central sensitization) [2], systemic low-grade inflammation, and muscle dysfunction [3–5]. These central and peripheral changes often occur concomitantly with clinical symptoms, such as depression [6] and sleep disturbance [7], which may compromise the biological rhythms. Consequently, it may also lead to a decrease in physical function, modifying the quality of life [3].

Brain-derived neurotrophic factor (BDNF) is a key molecule involved in plastic changes related to central and peripheral plasticity, neuroinflammation, pain, and other clinical symptoms in pathological conditions including FMS [1, 8]. Of note, FMS has a vastly negative impact on clinical and functional aspects, and current literature points to physical exercise and cognitive-behavioral therapy as the nonpharmacological choice interventions [9]. Once some interventions like exercise enhance the expression of BDNF in normal and pathological conditions, it is crucial to evaluate the efficacy of complementary therapeutic interventions on BDNF levels in FMS.

Unfortunately, evidence-supporting therapies for the management of FMS are limited to small trials of low methodological quality [10]. Mascarenhas et al., in a recent review, found moderate-quality evidence of a positive association between pain-reduction exercises and improved quality of life. The authors suggested that further high-quality trials might increase certainty with respect to the effectiveness of exercises in FMS [10].

Concerning exercises on the vibrating platform, a review work pointed out that whole-body vibration (WBV) exercises are safe, viable, and well tolerated by patients with chronic conditions including FMS and are less tiring and time-consuming than a standard exercise protocol [11]. In this regard, despite works showing WBV in fatigue and pain [9, 12], quality of life [9, 13–15], balance [9, 15–17], muscle strength [14], inflammatory status [4], and parameters of oxidative balance [18] in FMS patients, the works differed in aspects such as the vibratory stimulus (vertical or alternating), the vibratory protocol (frequency, amplitude, time of sets, rest interval, and duration), and time points (immediate or training) [19, 20]. Moreover, because FMS presents a negative influence on several outcomes (clinical, functional, and physiological) [10], there remains a gap regarding the evaluation of primary and secondary outcomes representing different aspects of the syndrome. In addition, the results of the works often present low effect size estimates, emphasizing the need for new studies with an experimental design and internal control ensuring methodological quality to fulfill the gaps that still exist [10]. Of note, the majority of previous works investigated the additional effects of the intervention combining whole-body vibration training (WBVT) with an associated exercise program, resulting in a gap regarding the stand-alone intervention effect [9]. Finally, as far as we know, no previous study evaluated the effects of WBVT on blood BDNF levels and crucial clinical (e.g., sleep quality and depression screening) symptoms associated with the biological rhythms in women with FMS. Therefore, our work aims to investigate the efficacy of WBVT on blood BDNF levels, clinical and functional outcomes, and quality of life in women with FMS. We hypothesize that stand-alone WBVT can promote changes in blood BDNF levels while improving lower limb muscle strength, aerobic capacity, clinical symptoms, sleep quality, and depressive symptoms.

## 2. Materials and Methods

### 2.1. Study Design

This was a randomized controlled clinical trial with concealed allocation and assessor blinding for score counts, developed at Universidade Federal dos Vales do Jequitinhonha e Mucuri (Federal University of the Jequitinhonha and Mucuri Valleys) (Diamantina/Minas Gerais, Brazil). This is a convenience sample. The recruitment of the patients was from health centers in the local community between June 2017 and June 2018. Randomization was performed using individual allocation code numbers placed within opaque, sealed envelopes, without contact with the participants.

The study was approved by the local ethics committee (identification number: 2.057.949) and registered on the Brazilian Clinical Trials Registry (REBEC; RBR-38nbbx). This study follows checklists for randomized and controlled clinical trials—Consolidated Standards of Reporting Trials (CONSORT) and Standard Protocol Items: Recommendations for Interventional Trials (SPIRIT).

### 2.2. Study Population

The inclusion criteria were being female, aged 50 to 60 years, from the perimenopause period onwards, and with a diagnosis of FMS confirmed by a rheumatologist. In addition, the patients also needed to be non-smokers and non-consumers of alcohol and be physically inactive, not having participated in any exercise programs during the previous 24 months. We highlight that the patients that self-reported physical activity levels lower than those recommended by the American College of Sports Medicine (ACSM) were classified as sedentary and were included [21].

The exclusion criteria were the presence of any concomitant disease that could be exacerbated by physical activity; inflammatory diseases; patients in psychiatric follow-up; patients performing physical activity more than twice a week; patients who displayed any of the possible contraindications for WBV stimulus, such as acute hernia, orthopedic and prosthetic lesions, metabolic or neuromuscular diseases, epilepsy, or stroke [22]; and patients taking oral or topical immunosuppressive medication (corticosteroids) [4]. The same requirements were applied to both groups.

Potential participants were screened to verify eligibility before baseline assessment and randomization. Only one researcher assigned the allocation of all the patients into the groups. All patients were asked which medications they were taking regularly (Table 1) and were randomly allocated to the intervention group (IG), who underwent WBVT, or the control group (CG), who did not receive the intervention. The IG patients underwent familiarization with the WBV stimulus and were informed as to the correct positioning and method of performing the exercise. CG patients received weekly phone calls from researcher and were instructed to maintain their routine of daily living activities. Follow-up occurred for the assessment of possible complications or changes in the daily routine, such as the presence of exacerbations, or the beginning of physical therapy or regular physical activity.

Both groups carried out baseline evaluations and follow-up after six weeks. In the IG, the second evaluation was performed 48 hours after the final intervention to minimize the residual effects of the final exercise session [12]. The evaluations always followed the same order. The participants came to the laboratory at 7 am having fasted for at least 8 hours and without using the medication they normally take in the morning. Moreover, all patients abstained from medication for at least 12 hours before evaluation to minimize possible acute effects. They were instructed to bring the medication to the laboratory. Soon after blood collection had been carried out, a standardized snack was offered, and the medication was ingested. Initially, personal and sociodemographic data were collected on the evaluation form, in addition to complete medical history, medications in use, and information on living habits. Blood collection was performed by a specialized professional and questionnaires were applied. Subsequently, functional tests and anthropometric assessments were performed.

### 2.3. Intervention

The IG performed WBVT three times per week on alternate days, for 6 weeks. The training protocol consisted of dynamic squatting, i.e., flexing lower limb joints during squatting for 3 seconds up, followed by 3 seconds down, on a synchronic vibrating platform (FitVibe® Excel Pro, GymnaUniphy, Belgium). The number of each set increased progressively over the 6 weeks. Thus, the patients performed sets of 6 to 8 squats. During each squat, the examiner instructed the patient to perform a semicomplete knee extension, i.e., up (angle 10°) for 3 seconds, followed by 3 seconds of knee bend, i.e., down (angle 60°). Although each squat required 6 seconds, because each position change (up/down-down/up) required 1 second, the total time of each squat was 8 seconds. Between sets, the patient was instructed to rest for 30 seconds on the vibratory platform turned off. Of note, each training day lasted around 180 to 624 seconds (i.e., 3 minutes to 10.6 minutes). To minimize resonant catastrophe, the participants were also instructed to remain with their feet on the platform and their spine, arms, and head in the instructed position (simulating the motion of sitting in a chair) [23]. The damping effect of different footwear was avoided through patients performing the exercises barefoot [24]. In addition, to ensure that each of the lower limbs received the same amount of vibration stimulus, a predetermined distance between the feet was set, with 14 cm to the right and 14 cm to the left of the platform vibration centre [25].

The mechanical stimulation parameters of the vibration consisted of the following: frequency of 35–40 Hz, amplitude of 4 mm, and acceleration gravity ranging from 2.78 to 3.26 g (Table 2). The training protocol was adapted from previous studies by our research group [4, 22, 26, 27]. A physical therapist monitored all the training sessions, including pain intensity and perceived exertion (RPE) before and after each intervention session. Of note, although pain and RPE were assessed during the exercise sessions (study internal control), we did not find any difference between subjects before and after the sessions while the intervention progressed.

### 2.4. Outcome Measures

#### 2.4.1. Primary Outcomes: Measurement of Blood BDNF Levels

Peripheral blood samples were collected aseptically by puncturing the median cubital vein. Blood was collected with the patient at rest for at least 10 minutes. The blood sample was then centrifuged twice at 3000 rpm for 10 minutes. The plasma was kept frozen at −80 °C until blood analyses. Blood BDNF levels were measured using a conventional sandwich enzyme-linked immunosorbent assay kit (DuoSet, R&D Systems, Minneapolis, MN, USA), according to the manufacturer's instructions. The detection limit was 5.0 pg/mL for the kit.

#### 2.4.2. Secondary Outcomes: Lower Limb Muscle Strength, Aerobic Capacity, Quality of Life, and Clinical Symptoms

The sit-to-stand test (STS) was used to assess lower limb muscle strength [28], and aerobic capacity was assessed using the 6-minute walk test (6MWT) [29, 30]. The Brazilian version of the Fibromyalgia Impact Questionnaire (FIQ) was used to assess health status, functional capacity, and main symptoms of FMS [31]. Quality of sleep, depression, and pain intensity were assessed using the Pittsburgh Sleep Quality Index (PSQI) [32], the Beck Depression Inventory [33], and the visual analogue scale (VAS) [34], respectively. The assessor was previously trained, and the intra-assessor reliability was greater than 80% for all outcomes. In addition, the same blinded assessor collected all the secondary outcomes [4].

### 2.5. Statistical Analysis

The data were reported as mean and 95% confidence interval (CI). For each outcome variable, we used a two-way repeated measure ANOVA to compare the main effects over time (time effect) and the interaction (group × time interactions). Post hoc analyses were evaluated using the Scheffé test. The level of statistical significance was set to *p* < 0.05. Effect size (eta squared: *ƞ*2) < 0.25 represented small effect, between 0.25 and 0.4 represented moderate effect, and >0.4 represented large effect [35]. The statistical power was also determined. As there were no missing data, intention-to-treat analyses were not performed.

The sample size to produce a significant effect was estimated at 15 volunteers per group, considering the comparison between groups for the blood BDNF levels (primary outcome), with an effect size of 1.1, statistical power of 80%, and alpha error of 5% [26].

## 3. Results

In total, 71 patients were screened for eligibility. Of these, 36 did not meet the inclusion criteria and 3 refused to participate. Thus, 32 women with FMS participated in the study and were randomized into two groups, that is, 17 patients in the IG and 15 in the CG (Figure 1).

At the baseline, there were no significant differences between the groups in patient characteristics. Patients from the CG and the IG were overweight according to the body mass index (BMI) classification (29.79 + 3.10 and 29.88 + 4.59 kg/m2, respectively) (Table 3).

There was no statistical difference between the groups regarding the blood BDNF levels or clinical and functional outcomes at baseline (Table 4).

There was an interaction effect (group-by-time) after the WBVT (Table 5 and Figure 2). IG patients showed increased blood BDNF levels (*p*=0.045), a higher number of repetitions on the STS test (*p*=0.011), and increased walking distance on the 6MWT (*p*=0.010) compared to the CG. There was also a decrease in scores on the FIQ (*p*=0.001), the PSQI (*p*=0.001), and the BDI (*p*=0.017) questionnaires and in the perception of pain assessed using VAS (*p*=0.008).

## 4. Discussion

To the best of our knowledge, this study is the first to evaluate the WBVT effect on blood BDNF levels and symptoms associated to the biological rhythms (e.g., sleep quality and depression screening) in women with FMS. The major findings demonstrated the following: (i) increased blood BDNF levels; (ii) improved lower limb muscle strength and aerobic capacity; (iii) improved clinical symptoms, i.e., sleep quality, depression symptoms, pain; and (iv) improved quality of life after a 6-week intervention of WBVT.

FMS symptoms are often related to physical inactivity, which in turn contributes and reinforces the impact of FMS, compromising physical activity, limiting daily function, and leading to progressive deconditioning with further reductions in physical capacity in FMS patients [36, 37]. Therefore, the results of improved physical function and exercise capacity after WBVT are clinically important evidencing the positive stand-alone effect of WBVT in physical aspects of FMS patients. In addition, the FIQ score reduction is of great clinical relevance demonstrating that stand-alone WBVT also promotes improvement in health status, functional capacity, and the main FMS symptoms, i.e., pain and fatigue, thereby reducing the impact of the disease and promoting an improvement in quality of life [38].

The literature demonstrates that plasma-free BDNF represents only the free (unbound) portion. This small fraction of unbound BDNF represents the bioavailable pool free to associate with TrkB or p75 receptors [39]. Thus, the WBVT probably promoted an increase in the BDNF portion while also reducing pain. Thus, we believe that the increase in blood BDNF levels (which represents the free unbound portion) seems to indicate a chronic adaptation inherent to training, influencing the pain defense mechanism. In addition, we believe that there was the maintenance of BDNF levels to the circulating pool, including musculoskeletal tissue cells. This hypothesis is in line with studies that have demonstrated that BDNF is a protein acting in autocrine and/or paracrine signalling within skeletal muscle. The expression increases through muscle contraction to enhance fat oxidation in an AMPK-dependent manner [40, 41].

Because BDNF plays an important role in the pathophysiology of the stress response and the pathogenesis of stress-associated mood disorders and its restoration may represent a critical mechanism underlying the antidepressant therapeutic effects, many investigators have focused on BDNF as a probable biomarker in depression. This is because the protein can cross the blood-brain barrier and circulating BDNF was correspondingly associated with cortical BDNF levels [42, 43]. However, it is still unknown whether BDNF alters sleep quality [44].

Previous studies indicated a possible link between improvement in subjective sleep outcomes and pain reduction in patients with FMS [34, 45]. Of note, the role of sleep quality in controlling pain and the pathophysiology of FMS suggests the need to develop alternatives to improve sleep quality. Some hypotheses try to explain the mode of action of WBVT in pain reduction. For example, activation of A-fibers produced during vibration can compete with central and peripheral nociceptive activity in the dorsal horn of the spinal cord, resulting in reduced second-order nociceptive activity with a consequent decrease in pain perception [23].

Although our experimental design did not focus on investigating associations and disease impact on different outcomes that affect biological rhythms in FMS patients, previous works suggested an association between the variables investigated in our work in FMS patients [36, 46]. Our statistical analysis does not allow causal inferences about the relationships between our outcome variables. Thus, we cannot make the claim that the BDNF is responsible for any change in other outcome variables given our study design and analysis.

However, it is worthwhile to highlight the large effect size (greater than 0.8) for most the outcomes, and only the sleep quality showed a moderate effect size (0.38) [35]. With this respect, the size of our sample was adequate to estimate the effect size. Thus, our analysis showed the short-term effects of WBVT in FMS were also clinically important in addition to being statistically significant for the outcomes and instruments assessed.

Thus, we suggested as a perspective to carry out further studies investigating the associations between BDNF plasma levels and clinical and functional outcomes including mediation/moderation analyses to confirm the hypothesis.

We emphasize that our study is at the forefront because no previous study investigated WBVT as a stand-alone intervention to FMS patients considering outcomes that together modify biological rhythms.

## 5. Strengths and Limitations

We highlight as strength the methodological quality because our work obtained a score of 8 in 10 points in the Physiotherapy Evidence Database Scale (PEDro scale) [47]. It is noteworthy that the items not reached in the total score (blinding of the subjects and therapist who administered the therapy) do not apply to studies with WBVT.

Although patients in both groups were instructed to abstain from using medication for 12 hours before experimental procedures, the possible chronic effect of medication intake on blood BDNF levels cannot be excluded, especially that of antidepressants [48]. However, surprisingly, the use of antidepressants was more common in the CG.

Another limitation was that we only analysed blood BDNF levels as biomarker. Thus, despite the contribution of blood BDNF levels to the circulating total, they are considerably lower than those of serum, so this small fraction of unbound BDNF represents a bioavailable pool that is free to associate with TrkB or p75 receptors [39, 49]. Despite this, we observed group vs time interactions in BDNF levels.

The level of general social interaction may also account for the results, as the control group did not experience these social exchanges. However, the patients of the control group received weekly phone calls to minimize this aspect. Moreover, the fact that the level of physical activity was self-reported by the patients may also constitute a limitation of the study.

Finally, our results cannot be generalized to other populations (e.g., different gender and age groups), as blood BDNF levels seem to interact with age and menstrual cycle.

## 6. Conclusions

Our data together are clinically relevant demonstrating the efficacy of WBVT maintaining blood BDNF levels with concomitant improvement in aspects related to biological rhythm (i.e., quality of sleep and depression symptoms). In addition, our data reinforced the WBVT effectiveness in reducing pain intensity and improving lower limb muscle strength, aerobic capacity, and quality of life in women with FMS.

## Figures and Tables

**Figure 1:** CONSORT flow diagram for the study.

**Figure 2:** Group x time effect of blood BDNF level, clinical and functional symptoms at baseline and 6-week follow-up. Blue represents the control group (CG, *n* = 15), and red represents the intervention group (IG, *n* = 17). The results are presented as mean ± SEM. (a) Blood brain-derived neurotrophic factor (BDNF) levels. (b) Sit-to-stand test (STS), rep (repetitions). (c) Six-minute walk test (6MWT). (d) Fibromyalgia Impact Questionnaire (FIQ). (e) Sleep quality: Pittsburgh Sleep Quality Index (PSQI). (f) Depression screening: Beck Depression Inventory (BDI). (g) Pain: visual analogue scale (VAS). Means followed by different symbols (^*∗*^) represent significance within group (time effect). Means followed by different lowercase letters (a, b) represent significance between groups (group × time interactions) (Scheffé test, *p* < 0.05).

**Table 1:** Medications of the patients.

Medication	CG (*n* = 15)	IG (*n* = 17)
Gastric distress	1 (6.6%)	2 (11.7%)
Analgesics	2 (13.3%)	7 (41.1%)
Anticonvulsant	2 (13.3%)	4 (23.5%)
Antidepressants	10 (66.6%)	6 (35.2%)
Antidiabetic	5 (33.3%)	3 (17.6%)
Antihypertensive	9 (60%)	5 (29.4%)
Anxiolytics	2 (13.3%)	0 (0.0%)
Antirheumatic	1 (6.6%)	1 (5.8%)
Neuropathic pain	2 (13.3%)	2 (11.7%)
Hypercholesterolemia	2 (13.3%)	4 (23.5%)
TSH suppression	2 (13.3%)	2 (11.7%)
Muscle relaxants	2 (13.3%)	2 (11.7%)

The numbers represent the number and percentage of participants in the group who use the medication. CG: control group (*n* = 15). IG: intervention group (*n* = 17).

**Table 2:** Whole-body vibration training load program (adapted from [22]).

Weeks	Vibration parameters (intervention group)			Total time per set (sec)	Number of repetitions per set	Total number of sets	Rest time between sets (seconds)
	Frequency (Hz)	Amplitude (mm)	Acceleration (G)				
1	35	4	2.78	16	5	6	30
2	35	4	2.78	24	8	7	30
3	35	4	2.78	32	10	8	30
4	40	4	3.26	35	11	8	30
5	40	4	3.26	40	13	8	30
6	40	4	3.26	48	16	8	30

Hz: hertz; mm: millimetres; G: gravity acceleration.

**Table 3:** Demographic, clinical, and anthropometric characteristics at baseline.

Outcome	CG (*n* = 15)	IG (*n* = 17)	*p* value
Age (years)	54 (50–58)	56 (53–59)	0.426
Time since diagnosis (years)	7.67 (5.73–9.61)	9.53 (7.46–11.60)	0.183
Weight (kg)	71.35 (66.79–75.91)	72.09 (65.64–78.52)	0.849
Height (m)	1.56 (1.53–1.59)	1.56 (1.54–1.58)	0.839
BMI (kg/m^2^)	29.79 (28.07–31.51)	29.88 (27.52–32.24)	0.953

Values are means (95% confidence interval). CG: control group (*n* = 15). IG: intervention group (*n* = 17). BMI: body mass index. *p* value: unpaired *t*-test.

**Table 4:** Biomarker levels and clinical and functional outcomes at baseline.

Outcome	CG (*n* = 15)	IG (*n* = 17)	*p* value
*Biomarker(ng/mL)*			
BDNF	2.39 (1.82–2.96)	2.35 (1.59–3.11)	0.922

*Functional outcomes*			
6MWT, m	427.27 (398.96–455.58)	447.35 (418.78–476.74)	0.292
STS, rep.	8.27 (6.71–9.93)	8.00 (6.48–9.52)	0.976

*Clinical outcomes*			
FIQ, score	66.68 (59.27–74.09)	72.53 (64.21–80.85)	0.277
Pain, VAS	5.77 (4.55–6.99)	7.14 (6.24–8.04)	0.081
PSQI, score	13.33 (11.61–15.05)	12.18 (9.78–14.58)	0.422
BDI, score	25.20 (19.34–31.06)	21.65 (16.43–26.87)	0.341

Values are means (95% confidence interval). CG: control group (*n* = 15). IG: intervention group (*n* = 17). BDNF, brain-derived neurotrophic factor; 6MWT, six-minute walk test; STS, sit-to-stand test; rep: repetition; FIQ, Fibromyalgia Impact Questionnaire; VAS, visual analogue scale; PSQI, Pittsburgh Sleep Quality Index; BDI, Beck Depression Inventory. *p* value: unpaired *t*-test (all variables showed normal distribution).

**Table 5:** Effects of 6 weeks of intervention and change from baseline on biomarker levels, functional outcomes, and clinical outcomes in control and whole-body vibration training groups.

Outcome	CG (week 6)	Δ (change from baseline)	IG (week 6)	Δ (change from baseline)	Interaction *p* value	Partial *η*^2^	Power
*Biomarker(ng/mL)*							
BDNF	1.80 (1.42 to 2.19)	−0.58 (−0.39 to −0.77)	2.58 (1.83 to 3.34)	0.23 (0.03 to 0.43)	**0.045**	0.81	0.99

*Functional outcomes*							
6MWT, m	415.40 (396.63 to 434.17)	−11.87 (−30.80 to 7.06)	470.35 (445.68 to 495.02)	22.59 (3.68 to 41.50)	**0.010**	0.88	1.0
STS, rep.	8.67 (7.22 to 10.12)	0.40 (−0.22 to 1.02)	10.41 (9.16 to 11.66)	2.41 (1.04 to 3.78)	**0.011**	0.88	1.0

*Clinical outcomes*							
FIQ, score	68.79 (62.23 to 75.35)	2.12 (−4.45 to 8.69)	45.12 (34.99 to 55.25)	−27.41 (−34.81 to 20.01)	**0.001**	0.97	1.0
Pain, VAS	5.91 (4.78 to 7.04)	0.15 (−1.44 to 1.74)	3.46 (2.06 to 4.86)	3.46 (2.06 to 4.86)	**0.008**	0.93	1.0
PSQI, score	14.13 (12.37 to 15.89)	0.80 (−0.64 to 2.24)	7.18 (5.18 to 9.18)	−5.00 (−7.04 to 2.96)	**0.001**	0.38	0.34
BDI, score	25.20 (19.40 to 31.00)	0 (−1.26 to 1.26)	14.76 (9.10 to 20.42)	−6.88 (−12.17 to −1.59)	**0.017**	0.86	1.0

Values are means (95% confidence interval). CG: control group (*n* = 15). IG: intervention group (*n* = 17). BDNF: brain-derived neurotrophic factor; 6MWT: six-minute walk test; STS: sit-to-stand test; rep.: repetition; FIQ: Fibromyalgia Impact Questionnaire; VAS: visual analog scale; PSQI: Pittsburgh Sleep Quality Index; BDI: Beck Depression Inventory. Interaction, group *x* time. Eta partial, *η*^2^.

## Data Availability

The study data are with the researchers and can be provided when necessary.

## References

[1] Theoharides T. C., Tsilioni I., Bawazeer M. (2019). Mast cells, neuroinflammation and pain in fibromyalgia syndrome. *Frontiers in Cellular Neuroscience*.

[2] Woolf C. J. (2011). Central sensitization: implications for the diagnosis and treatment of pain. *Pain*.

[3] Alciati A., Atzeni F., Grassi M. (2018). Features of mood associated with high body weight in females with fibromyalgia. *Comprehensive Psychiatry*.

[4] Ribeiro V., Mendonça V., Souza A. (2018). Inflammatory biomarkers responses after acute whole body vibration in fibromyalgia. *Brazilian Journal of Medical and Biological Research*.

[5] Jablochkova A., Bäckryd E., Kosek E. (2019). Unaltered low nerve growth factor and high brain-derived neurotrophic factor levels in plasma from patients with fibromyalgia after a 15-week progressive resistance exercise. *Journal of Rehabilitation Medicine*.

[6] Nugraha B., Karst M., Engeli S., Gutenbrunner C. (2012). Brain-derived neurotrophic factor and exercise in fibromyalgia syndrome patients: a mini review. *Rheumatology International*.

[7] Nijs J., Loggia M. L., Polli A. (2017). Sleep disturbances and severe stress as glial activators: key targets for treating central sensitization in chronic pain patients?. *Expert Opinion on Therapeutic Targets*.

[8] Bjersing J. L., Erlandsson M., Bokarewa M. I., Mannerkorpi K. (2013). Exercise and obesity in fibromyalgia: beneficial roles of IGF-1 and resistin?. *Arthritis Research & Therapy*.

[9] Mingorance JA, Montoya P, Miranda JGV, Riquelme I (2021). The Therapeutic Effects of Whole-Body Vibration in Patients With Fibromyalgia. A Randomized Controlled Trial. *Frontiers in Neurology*.

[10] Mascarenhas R. O., Souza M. B., Oliveira M. X. (2020). Association of therapies with reduced pain and improved quality of life in patients with fibromyalgia: a systematic review and meta-analysis. *JAMA Internal Medicine*.

[11] Stania M., Juras G., Słomka K., Chmielewska D., Król P. (2016). The application of whole-body vibration in physiotherapy - A narrative review. *Acta Physiologica Hungarica*.

[12] Alentorn-Geli E., Padilla J., Moras G., Haro C. L., Fernández-Solà J. (2008). Six weeks of whole-body vibration exercise improves pain and fatigue in women with fibromyalgia. *The Journal of Alternative and Complementary Medicine*.

[13] Olivares P. R., Gusi N., Parraca J. A., Adsuar J. C., Del Pozo-Cruz B. (2011). Tilting whole body vibration improves quality of life in women with fibromyalgia: a randomized controlled trial. *The Journal of Alternative and Complementary Medicine*.

[14] Sañudo Corrales FdB, Hoyo Lora Md, Carrasco Páez L., McVeigh JG, Corral Pernia JA, Cabeza Ruiz R (2010). The effect of a 6-week exercise programme and whole body vibration on strength and quality of life in women with fibromyalgia: a randomised study. *Clinical and Experimental Rheumatology*.

[15] Sañudo B., Carrasco L., Hoyo M., Oliva-Pascual-Vaca C, Rodríguez-Blanco C. (2013). Changes in body balance and functional performance following whole-body vibration training in patients with fibromyalgia syndrome: A randomized controlled trial. *Journal of rehabilitation medicine*.

[16] Adsuar J, Del Pozo-Cruz B, Parraca J, Olivares P, Gusi N (2012). The single-leg stance static balance in women with fibromyalgia: A randomized controlled trial. *The Journal of sports medicine and physical fitness*.

[17] Sañudo B., de Hoyo M., Carrasco L., Rodríguez-Blanco C., Oliva-Pascual-Vaca Á., McVeigh J. G. (2012). Effect of whole-body vibration exercise on balance in women with fibromyalgia syndrome: a randomized controlled trial. *The Journal of Alternative and Complementary Medicine*.

[18] Santos J, Mendonça V, Ribeiro V, Tossige-Gomes R, Fonseca S, Prates A (2019). Does whole body vibration exercise improve oxidative stress markers in women with fibromyalgia?. *Brazilian Journal of Medical and Biological Research*.

[19] Bidonde J., Busch A. J., van der Spuy I., Tupper S., Kim S. Y., Boden C. (2017). Whole body vibration exercise training for fibromyalgia. *Cochrane Database of Systematic Reviews*.

[20] Dong Y., Wang W., Zheng J., Chen S., Qiao J., Wang X. (2019). Whole body vibration exercise for chronic musculoskeletal pain: a systematic review and meta-analysis of randomized controlled trials. *Archives of Physical Medicine and Rehabilitation*.

[21] WHO (2020). *Guidelines on Physical Activity and Sedentary Behaviour*.

[22] Avelar N. C. P., Simão A. P., Tossige-Gomes R. (2011). The effect of adding whole-body vibration to squat training on the functional performance and self-report of disease status in elderly patients with knee osteoarthritis: a randomized, controlled clinical study. *The Journal of Alternative and Complementary Medicine*.

[23] Rittweger J. (2010). Vibration as an exercise modality: how it may work, and what its potential might be. *European Journal of Applied Physiology*.

[24] Marín P. J., Bunker D., Rhea M. R., Ayllón F. N. (2009). Neuromuscular activity during whole-body vibration of different amplitudes and footwear conditions: implications for prescription of vibratory stimulation. *Journal of Strength and Conditioning Research*.

[25] Simão A. P., Avelar N. C., Tossige-Gomes R. (2012). Functional performance and inflammatory cytokines after squat exercises and whole-body vibration in elderly individuals with knee osteoarthritis. *Archives of Physical Medicine and Rehabilitation*.

[26] Simão AP, Mendonça VA, Avelar NCP (2019). Whole Body Vibration Training on Muscle Strength and Brain-Derived Neurotrophic Factor Levels in Elderly Woman with Knee Osteoarthritis: A Randomized Clinical Trial Study. *Frontiers in physiology*.

[27] Neves C. D. C., Lacerda A. C. R., Lage V. K. S. (2018). Whole body vibration training increases physical measures and quality of life without altering inflammatory-oxidative biomarkers in patients with moderate COPD. *Journal of Applied Physiology*.

[28] Collado-Mateo D., Adsuar J. C., Dominguez-Muñoz F. J., Olivares P. R., Gusi N. (2017). Impact of fibromyalgia in the sit-to-stand-to-sit performance compared with healthy controls. *PM&R*.

[29] ATS Committee on Proficiency Standards for Clinical Pulmonary Function Laboratories (2002). ATS statement: guidelines for the six-minute walk test. *American Journal of Respiratory and Critical Care Medicine*.

[30] Mannerkorpi K., Svantesson U., Carlsson J., Ekdahl C. (1999). Tests of functional limitations in fibromyalgia syndrome: a reliability study. *Arthritis & Rheumatism*.

[31] Marques A. P., Santos A. M. B., Assumpção A., Matsutani L. A., Lage L. V., Pereira C. A. B. (2006). Validação da versão bra-sileira do Fibromyalgia Impact Questionnaire (FIQ). *Revista Brasileira de Reumatologia*.

[32] Bertolazi A. N., Fagondes S. C., Hoff L. S. (2011). Validation of the Brazilian Portuguese version of the Pittsburgh sleep quality index. *Sleep Medicine*.

[33] Gomes-Oliveira M. H., Gorenstein C., Neto F. L., Andrade L. H., Wang Y. P. (2012). Validation of the Brazilian Portuguese version of the Beck Depression Inventory-II in a community sample. *Revista Brasileira de Psiquiatria*.

[34] Bigatti S. M., Cronan T. A. (2002). A comparison of pain measures used with patients with fibromyalgia. *Journal of Nursing Measurement*.

[35] Cohen J. (1973). Eta-squared and partial eta-squared in fixed factor ANOVA designs. *Educational and Psychological Measurement*.

[36] Assumpção A, Sauer JF, Mango PC, Pascual Marques A (2010). Physical function interfering with pain and symptoms in fibromyalgia patients. *Clinical and experimental rheumatology*.

[37] Gaudreault N., Boulay P. (2018). Cardiorespiratory fitness among adults with fibromyalgia. *Breathe*.

[38] Williams DA, Arnold LM (2011). Measures Applied to the Assessment of Fibromyalgia: Fibromyalgia Impact Questionnaire (FIQ), Brief Pain Inventory (BPI), the Multidimensional Fatigue Inventory (MFI-20), the MOS Sleep Scale, and the Multiple Ability Self-Report Questionnaire (MASQ; cognitive dysfunction). *Arthritis Care & Research*.

[39] Walsh J. J., Tschakovsky M. E. (2018). Exercise and circulating BDNF: mechanisms of release and implications for the design of exercise interventions. *Applied Physiology, Nutrition, and Metabolism*.

[40] Bogaerts A., Delecluse C., Claessens A. L., Coudyzer W., Boonen S., Verschueren S. M. P. (2007). Impact of whole-body vibration training versus fitness training on muscle strength and muscle mass in older men: a 1-year randomized controlled trial. *The Journals of Gerontology Series A: Biological Sciences and Medical Sciences*.

[41] Krabbe K. S., Mortensen E. L., Avlund K. (2009). Brain-Derived Neurotrophic Factor Predicts Mortality Risk in Older Women. *Journal of the American Geriatrics Society*.

[42] Schmitt K., Holsboer-Trachsler E., Eckert A. (2016). BDNF in sleep, insomnia, and sleep deprivation. *Annals of Medicine*.

[43] Karege F., Perret G., Bondolfi G., Schwald M., Bertschy G., Aubry J.-M. (2002). Decreased serum brain-derived neurotrophic factor levels in major depressed patients. *Psychiatry Research*.

[44] Uchida S., Shioda K., Morita Y., Kubota C., Ganeko M., Takeda N. (2012). Exercise effects on sleep physiology. *Frontiers in Neurology*.

[45] Çetin B., Güleç H., Toktaş H. E., Ulutaş Ö., Yılmaz S. G., İsbir T. (2018). Objective measures of sleep in fibromyalgia syndrome: Relationship to clinical, psychiatric, and immunological variables. *Psychiatry Research*.

[46] Häuser W (2016). Fibromyalgia syndrome: Basic knowledge, diagnosis and treatment. *Medizinische Monatsschrift fur Pharmazeuten*.

[47] Blobaum P (2006). Physiotherapy evidence database (PEDro). *Journal of the Medical Library Association*.

[48] Sumpton J. E., Moulin D. E. (2008). Fibromyalgia: presentation and management with a focus on pharmacological treatment. *Pain Research and Management*.

[49] Zagrebelsky M., Korte M. (2014). Form follows function: BDNF and its involvement in sculpting the function and structure of synapses. *Neuropharmacology*.

